# Germacrone exerts anti-cancer effects on gastric cancer through induction of cell cycle arrest and promotion of apoptosis

**DOI:** 10.1186/s12906-019-2810-3

**Published:** 2020-01-23

**Authors:** Lei Wu, Lifen Wang, Xiangguo Tian, Junyong Zhang, Hua Feng

**Affiliations:** Department of Digestive Disease, Shandong Provincial Hospital Affiliated to Shandong University, No. 324, the Five Weft Seven Road, Ji’nan City, Shandong Province 250021 People’s Republic of China

**Keywords:** Germacrone, Cell cycle arrest, Apoptosis, Gastric cancer, BGC823 cells

## Abstract

**Background:**

Germacrone is one of the natural bioactive compounds found in *Rhizoma curcuma* essential oils. In this study, the potential anti-cancer effect of germacrone in gastric cancer cell line BGC823 was investigated.

**Methods:**

The cell viability and proliferative activity were assessed, and cell cycle analysis was also performed. Hoechst 33258 and Annexin V/PI double staining was used for detection of cell apoptosis. Protein profiles of cell cycle-related and apoptosis-related proteins were assessed.

**Results:**

MTT assay revealed that germacrone had marked cytotoxicity on BGC823 cells. Germacrone induced cell cycle arrest in the G2/M phase via remarkably decreased expression levels of cyclin B1, cdc 2 and cdc 25c. In addition, the treatment with germacrone induced caspase-3 activity and PARP cleavage. These findings demonstrated the effects of germacrone on inhibiting cell proliferation through induction of G2/M phase cell cycle arrest and promotion of cell apoptosis. It also indicated that germacrone functioned through modulations of cell cycle-associated protein expression and mitochondria-mediated apoptosis.

**Conclusion:**

These findings will be valuable as the molecular basis for the germacrone-mediated anti-cancer effect against gastric cancer.

## Background

Gastric cancer is a frequently occurring malignant cancer type and a leading cause of cancer death globally, especially in some Asian countries like China and Japan [1, 2]. Gastric cancer usually has delayed symptoms, so patients usually already developed into advanced stages of metastasis when diagnosed [3]. The main clinical treatments for gastric cancer often include surgical operation, radiation therapy and chemotherapy. Although for many cases the treatments are effective, the high morbidity rate and low 5-year survival rate of gastric cancer make it a serious health risk [4]. Therefore, more effective therapeutic approaches are of great importance for the prognosis of gastric cancer patients.

Traditional Chinese herbs serving as successful therapeutic drugs in the treatment of different types of cancers have been proved [5]. *Rhizoma curcuma*, a traditional Chinese herbal medicine, is commonly prescribed for treating inflammation and cancer therapy [6]. Many essential oils of *Rhizoma curcuma* are the principal bioactive constituents that have anti-inflammatory and anti-tumor properties [7, 8]. Germacrone is a natural bioactive compound found in *Rhizoma curcuma* essential oils [9, 10]. Studies on the biological activities of germacrone have demonstrated that it also possesses significant protective effects including anti-bacterial, anti-fungal, antifeedant, depressant, choleretic, antitussive and vasodilator activities [11–14]. These findings lead to the hypothesis in this study that germacrone might be involved in anti-tumor effect in human gastric cancer.

Cell cycle arrest is an essential regulatory mechanism in cell proliferation and tumor development. A typical feature of cancer cells is the aperiodicity of cell cycle. DNA damage in the cells can activate the repairing system and many signal transduction pathways, which result in cell cycle arrest and apoptosis [15]. G2/M phase is a major cell cycle checkpoint in cancer treatment because it allows the cells containing damaged DNA to repair the damage at the G2/M checkpoint [16]. Germacrone has been reported to induce G0/G1 or G2/M phase cell cycle arrest in various cancer cell lines [13]. Variations of cell cycle regulation in different types of cancer cells might due to differences associated with cell type [17]. It is well studied that cyclin proteins play important roles in regulating cell cycle process [18]. Cyclin B1, cell division cyclin 2 (cdc2) and cdc 25 are crucial regulators associated with the G2 to M phase transition [19].

Apoptosis is another core regulator of cell proliferation and cell death, which makes it a major factor that is targeted for cancer therapy. In the process of apoptosis, caspases function by executing cell death through different apoptotic stimuli [20, 21]. The distinct roles of caspase family members in cell apoptosis have been widely reported. Caspases associated with apoptosis have been classified based on their functions into the initiator, inhibitor and inflammatory caspases [22, 23]. The regulation of caspase activation involves in different cellular proteins including Bcl-2 protein family, which is known to be involved in the mitochondrial apoptosis pathway. They are classified into two groups as the pro-apoptotic (Bax, Bak) and anti-apoptotic (Bcl-2, Bcl-xl, Bcl-w, Mcl-1) proteins [24, 25]. Bax/Bcl-xl ratio is demonstrated to be highly associated with the extent of apoptosis [26].

Here, the anti-cancer effect of germacrone and underlying mechanisms of its activity were investigated in human gastric cancer cell line BGC823. Changes of cell cycle arrest and apoptosis after germacrone treatment were assessed, and potential mechanisms were explored. Our findings will have valuable perception on the germacrone-mediated anti-cancer effect against gastric cancer.

## Methods

### Cell line and morphological assessment

Human gastric cancer BGC823 cells (obtained from Cell Research Institute of the Chinese Academy of Science) were cultured in RPMI-1640 medium supplemented with 10% FBS, 100 μg/mL penicillin and 100 μg/mL streptomycin in a humidified incubator at 37 °C with 5% CO_2_. Germacrone (Chengdu MUST Bio-technology CO., LTD, Chengdu, China) in serial concentrations as dissolved in DMSO (20, 40, 60, 80 μM) were added to the culture medium. DMSO (0 μM germacrone) was used as control. After incubation for 6, 12, 18, 24 and 48 h, cell morphological changes were monitored through an inverted microscope (Zeiss Axio Observer A1).

### Cell viability assessment using MTT assay

BGC823 cells were seeded into 96-well plate (5 × 10^3^) and were incubated for 24 h. Germacrone in serial concentrations as dissolved in DMSO (20, 40, 60, and 80 μM) were added to the cells. DMSO (0 μM germacrone) was used as control. After 12, 24, 48 and 72 h of germacrone treatment, 50 μg MTT was added and cells were incubated in dark at 37 °C for 4 h. The MTT-containing medium was discarded and the formazan product was dissolved by adding 100 μl of DMSO. The solution was shaking for 10 min in dark and the absorbance value was measured at the wavelength of 570 nm with a Multiskan Spectrum Microplate Reader (Thermo, USA).

### Cell cycle assessment

BGC823 cells were synchronized in serum-free medium for 24 h and then treated with DMSO or in serial concentrations of germacrone (20, 40, 60, and 80 μM) at 37 °C for 24 h, followed by washing with phosphate buffered saline (PBS) twice. Cells were trypsinized and collected by centrifugation, followed by fixation in 70% ethanol at 4 °C for 24 h. After washing with PBS, cells were stained by propidium iodide (PI) in staining solution supplemented with RNase A for 30 min. Cell cycle was assessed using the FACScan flow cytometer. Data were analyzed with the CellQuest software.

### Apoptosis assay by Hoechst 33258 staining

BGC823 cells that were seeded into 12-well plates were incubated with germacrone in serial concentrations (20, 40, 60, 80 μM) at 37 °C for 24 h. After washing twice with PBS, cells were fixed in 3.7% paraformaldehyde solution for 15 min. The fixing solution was discarded, followed by staining with 5 μg/mL Hoechst 33258 for 10 min. Apoptotic cells were then assessed through a Leica fluorescence microscopy at 1000x magnification.

### Apoptosis assay by flow cytometry

The Fluorescein Isothiocyanate (FITC) Annexin V Apoptosis Detection Kit I (BD Pharmingen, San Diego, CA, USA) was used to detect apoptotic cells following the manufacturer’s protocol. In summary, BGC823 cells were treated with germacrone in serial concentrations (20, 40, 60, and 80 μM) at 37 °C for 24 h. After washing with PBS, cells were trypsinized and subsequently incubated in FITC-conjugated Annexin-V binding buffer containing PI in dark for 15 min. After incubation, cell apoptosis was assessed using a FACScan flow cytometer.

### Caspase-3, − 6, − 8 and − 9 activity assay

The protease activities of caspase-3, − 6, − 8 and − 9 in BGC823 cells were assessed using the Caspase Activation Kit (Millipore, Billerica, MA, USA) following the manufacture’s protocol. Briefly, BGC823 cells were resuspended in cell lysis buffer. After 15 min incubation, the supernatant of cell lysates was collected by centrifugation. Total proteins of cell extract were incubated with the mixture of caspase assay buffer and the corresponding caspase substrate specific for caspase-3, − 6, − 8 and − 9 at 37 °C for 1 h. The enzyme-linked optical density of the solution was measured by the immunosorbent assay at 405 nm wavelength with a spectrocolorimeter.

### Western blot

Equal amount of each protein sample was transferred to SDS-PAGE (12%) and then transferred to 0.45 mm PVDF membranes (Merck, Darmstadt, Germany), followed by blocking with TBST containing 5% skim milk for 1 h, and subsequent incubation with the corresponding primary antibody (1:1000, Cell Signaling Technology, Danvers, Mass, USA) at 4 °C for overnight, followed by incubation with HRP-conjugated secondary antibody (1:2000, Santa Cruz Biotechnology, Santa Cruz, CA, USA) for 2 h. Protein signals were detected by the enhanced chemiluminescence (ECL) assay. The Image J (NIH) software was used for quantification of proteins that were normalized relative to β-actin.

### Statistical analysis

Data values were presented as the mean ± standard deviation (SD) of three independent experiments. Significant difference for multiple-group comparison was performed by ANOVA analysis. Statistically significant difference was considered when *P* value < 0.05.

## Results

### Germacrone inhibits cell proliferation and viability of BGC823 cells

The changes caused by germacrone (chemical structure was shown in Fig. 1A) treatment on BGC823 cell morphology was observed under an optical microscopy at 200x magnification. Compared with the control group, in which cells without germacrone treatment exhibited normal morphology with well-shaped and orderly arrangement, the germacrone-treated cells (24 h) exhibited obvious morphological changes including shrunk, unclear shape, nuclear condensation, fewer number and disorderly arrangement of cells (Fig. 1B). All these morphological changes that are indicative of cell apoptotic death were observed with 12 h of treatment and became more remarkable as the increasing of germacrone concentration (20, 40, 60 and 80 μM) and treatment time (12, 24, 48 and 72 h) (data not shown). The MTT assay revealed that germacrone treatment significantly inhibited the growth of BGC823 cells and the degree of inhibition depends on both the concentration of germacrone and time of treatment (*P* < 0.05, *P* < 0.01) (Fig. 1C).

**Fig. 1:** Effect of germacrone on BGC823 cell proliferation and cell morphological changes. Cells were treated with germacrone at a serial of concentrations (0, 20, 40, 60, and 80 μM) for 12, 24, 48 and 72 h. **a** The chemical structure of germacrone. **b** Morphological observations BGC823 cells under optical microscopy at 200x magnification after 24 h treatment of germacrone in serial concentrations (0, 20, 40, 60, and 80 μM). **c** MTT assay showing the effect of germacrone on BGC823 cell proliferation cell. “*”: *P* < 0.05, “**”: *P* < 0.01

### Germacrone induced G2/M cell cycle arrest in gastric cancer cells

The effects of germacrone on cell cycle status of gastric cancer cells were assessed. The cell cycle distribution results showed that exposure of BGC823 cells to germacrone lead to a significant increase of cells at G2/M phase (*P* < 0.05, *P* < 0.01), while there was a significant decrease at S phase (*P* < 0.01) (Fig. 2). The percentage of BGC823 cells at the G2/M phase increased from 33.7 ± 1.22% (control) to 34.76 ± 0.75%, 35.98 ± 1.05%, 37.97 ± 1.66%, and 42.66 ± 2.06% after treatment with 20, 40, 60 and 80 μM of germacrone, respectively. And the percentage of BGC823 cells at S phase decreased from 29.4 ± 0.72% (control) to 27.81 ± 0.77%, 25.56 ± 0.66%, 22.9 ± 0.95%, 20.52 ± 0.63% after treated with 20, 40, 60 and 80 μM of germacrone, respectively. Cells at G0/G1 phase were not significantly changed after germacrone treatment (*P* > 0.05).

**Fig. 2:** Effect of germacrone on BGC823 cell cycle status. BGC823 cells were treated with germacrone with designated concentrations for 24 h. Flow cytometry analysis was performed to assess cell cycle phase status after staining with propidium iodide (PI). “*”: *P* < 0.05, “**”: *P* < 0.01

### Germacrone down-regulated the expression of cyclin B1, cdc 2 and cdc 25c

Protein expression profile was analyzed on three G2/M phase cell cycle-associated proteins including cyclin B1, cdc 2 and cdc 25c by Western blot. Germacrone treatment induced a decrease of the expression of cyclin B1, cdc 2, and cdc 25c, and the degree of decrease improved with the increasing of germacrone concentration (Fig. 3A). It showed a markedly decrease when germacrone concentrations were 60 and 80 μM (*P* < 0.05, *P* < 0.01) (Fig. 3B-D). These results indicated that germacrone-induced cell cycle arrest was associated with the downregulation of cyclin B1, cdc 2, and cdc 25c.

**Fig. 3:** Western blot analysis of cell cycle-associated proteins. Total proteins were prepared after BGC823 cells were treated with germacrone at different concentreations (0, 20, 40, 60, and 80 μM) and then analyzed by western blotting. **a** Representative blotting bend intensities used for the quantification of (**b**) protein cyclin B1, (**c**) protein cdc 2 and (**d**) protein cdc 25c. β-actin was used as an internal control. “*”: *P* < 0.05, “**”: *P* < 0.01

### Germacrone induced BGC823 cell apoptosis

The cell morphological changes observed after germacrone treatment were characteristic of cell apoptosis. To verify that germacrone can induce cell apoptosis, Hoechst staining and Annexin V-PI double staining were performed in BGC823 cells with 24 h treatment of germacrone at different concentrations (20, 40, 60 and 80 μM). As shown in Fig. 4A, compared with the cells without germacrone treatment, germacrone-treated cells had small and bright blue nuclei, which is indicative of cell apoptosis. Similarly, increasing dose of germacrone progressively increased cell apoptosis as indicated by the dose-dependent decrease of proportions of intact cells (Fig. 4B). These evidences proved that germacrone can induce apoptosis in BGC823 cells.

**Fig. 4:** Effect of germacrone on the induction of apoptosis in BGC823 cells. BGC823 cells were treated with germacrone for 24 h at different concentreations (0, 20, 40, 60, and 80 μM). **a** Neclear staining of BGC823 cells with Hoechst 33258. Cells were observed under fluorescence microscopy at 1000x magnification. **b** Annexin V-PI double staining assay detecting cell apoptosis. Percentages of early apoptotic cells (Annexin V staining) and necrotic apoptotic cells (both Annexin V-FITC and PI stainning) are shown

### Germacrone altered the expression of apoptosis-regulatory proteins

To further investigate the underlying mechanisms involved in germacrone-promoted apoptosis, expression levels of apoptosis-associated proteins were evaluated. Two mitochondria apoptosis-associated protein, Bcl-xL and Bax, were investigated. Western blot analysis showed that compared with cells without germacrone treatment, expression of pro-apoptotic protein Bax markedly up-regulated with the increase of germacrone concentration with a dose-dependent manner (Fig. 5A), whereas expression of anti-apoptotic protein Bcl-xL markedly down-regulated, with a dose-dependent manner as well. And the Bax/Bcl-xL ratio significantly increased when germacrone concentration is at 40, 60 and 80 μM (*P* < 0.05, *P* < 0.01) (Fig. 5B). Expressions of other apoptosis-related proteins were also assessed by western blot, including procaspase-3, − 6, − 8, − 9, cleaved PARP and cleaved caspase-3, − 6, − 8, − 9 (Fig. 6A). Compared with cells without germacrone treatment, the expression levels of procaspase-3, − 6, − 8, and − 9 gradually decreased with the increasing concentrations of germacrone (*P* < 0.05, *P* < 0.01) (Fig. 6B-E). The expression of cleaved PARP and cleaved caspase-3, − 6, − 8, − 9 increased dose-dependently with germacrone treatment (*P* < 0.01) (Fig. 6F). And the caspase-3 activities significantly increased after treating with germacrone (*P* < 0.05, *P* < 0.01) (Fig. 6G). These results indicated the effect of germacrone on inducing cell apoptosis by regulating the mitochondria apoptosis pathway and the caspase dependent pathway.

**Fig. 5:** Effect of germacrone on the expression of mitochondria apoptosis-regulatory proteins Bax and Bcl-xL. Total proteins were prepared after BGC823 cells were treated with germacrone at different concentreations (0, 20, 40, 60, and 80 μM) and then analyzed by western blotting. **a** Representative blotting bend intensities used for the quantification of Bax and Bcl-xL. **b** Quantitative data of the Bax/Bcl-xL ratio from protein expression. β-actin was used as an internal control. “*”: *P* < 0.05, “**”: *P* < 0.01

**Fig. 6:** Effect of germacrone on the expression of apoptosis-associated proteins procaspase**-**3, − 6, − 8, − 9, cleaved caspase-3, − 6, − 8, − 9**,** and cleaved PARP. Total proteins were prepared after BGC823 cells were treated with germacrone at different concentreations (0, 20, 40, 60, and 80 μM) and then analyzed by western blotting. **a** Representative blotting bend intensities of procaspase-3, − 6, − 8, − 9, cleaved caspase-3, − 6, − 8, − 9 and cleaved PARP that were used for quantification of protein procaspase-8 (**b**), protein procaspase-9 (**c**), protein procaspase-3 (**d**) protein procaspase-6 (**e**), and protein cleaved PARP (**f**) expressions. (**g**) Caspase-3 activity. β-actin was used as an internal control. “*”: *P* < 0.05, “**”: *P* < 0.01

## Discussions

Many traditional plant-derived medicinal herbs have been proved as effective and safe pharmaceutical compounds in cancer therapy, especially in Asian countries. The anti-cancer effect of germacrone, the component isolated from *Rhizoma curcuma*, was demonstrated in different cancer cells, including hepatocellular carcinoma, breast cancer, ovarian cancer, hepatoma and glioma [13, 27–29]. Here, the anti-cancer effect of germacrone was studied in gastric cancer cells. Viability assays revealed that germacrone could inhibit cell proliferation in the dose- and treatment time-dependent manner in BGC823 cells. As the anti-tumor capabilities of *Rhizoma curcuma* have been identified clinically in China [30], findings in the present study are inspiring for future studies on investigating the bioactivities of other volatile oil components isolated from *Rhizoma curcuma,* such as β-elemene, curcumol, curdione, neocurdione, etc.

Reduced cell proliferation resulted from cell cycle arrest is a typical feature in tumor suppression and has been widely demonstrated in different cancer cells. The G2/M checkpoint prevents cell cycle progression by repairing damaged DNA in the cell [16]. The induction of G2/M phase cell cycle arrest in suppressing cancer cell proliferation has been demonstrated in various cancer cells. For example, aloperine induces G2/M phase cell cycle arrest in human colon cancer cells [31], quercetin induces G2/M phase cell cycle arrest in human cervical cancer cells [32], and tetrahydroingenol diterpenoid induces G2/M phase cell cycle arrest in melanoma cancer cells [33]. Findings in the present study showed convincingly that germacrone inhibits cell proliferation in BGC823 cells by inducing G2/M phase arrest in the dose-dependent manner, while with a significant inhibition of the S phase. Lee et al. reported that similar to germacrone’s anti-cancer effect, flavonoids induced G2/M phase cell cycle arrest and cell apoptosis in human gastric cancer AGS cells [34]. In the cell cycle progression, cyclin B1, cdc 2, and cdc 25c are very influential proteins in the G2/M phase. Cyclin B1 and cdc 2 form a protein complex and regulate the transition from G2 to M phase. And cdc 25 regulates the protein complex formed between cyclin B and cdc 2 [19]. In the present study, germacrone down-regulated the expression of cyclin B1, cdc 2 and cdc 25c proteins, resulting in the suppression of BGC823 cell growth by inhibiting cell cycle progression in the G2/M phase. The activity of cyclinB1/cdc2 complex is regulated by many factors in G2/M transition, and down-regulation of cyclin B1 by germacrone observed in this study provided insights into the regulation of cell cycle progression. In addition to cyclins, cyclin-dependent kinases (cdks) are also important proteins in the cell cycle progression [18]. CDK2 has been identified as a key regulator of S phase cell cycle progression [35]. The cyclin E and cdk2 can form a protein complex and regulate cell cycle progression in late G1 phase. The cyclin D and cdk4/cdk6 form a complex to mediate cell cycle progression in the mid-G1 phase [36, 37]. The expressions of cdk proteins by the regulation of germacrone in BGC823 cells, which is not investigated in the present study, could be a promising point of view in further studies on the germacrone-regulated cell cycle progression in gastric cancer.

Apoptosis is a critical process in protecting organisms against abnormal growth by excluding cells that have been proliferated improperly. The Bcl-2 protein family contains key regulators that are involved in mitochondrial pathway-regulated apoptosis. Bcl-2 and Bcl-xL bind to mitochondria outer membrane to block the release of cytochrome *c* to the cytosol. The pro-apoptotic proteins Bax and Bak are essential for mitochondria outer membrane permeabilization during apoptosis [38, 39]. As expected, our results revealed that germacrone induced apoptosis of BGC823 cells. Germacrone treatment showed significant increase in the expression levels of pro-apoptotic Bax and significant decrease in the expression levels of anti-apoptotic Bcl-xL. Caspases play critical roles in apoptosis as well. The apoptosis resulted from germacrone treatment was matching with the morphological changes in BGC823 cells. Germacrone treatment resulted in down-regulation of procaspase-3, − 6, − 8, and − 9, which in turn induced the activity of cleaved caspase-3, − 6, − 8, and − 9, which are essential caspases in the regulation of apoptosis [40]. The enhanced activity of caspase-3 also induced the cleavage of poly-ADP-ribose polymerase (PARP), which is a distinguishing feature of caspase-dependent apoptosis [41].

This study emphasized on elucidating the function of germacrone in anti-proliferative and pro-apoptotic of BGC823 cells. However, except for cell proliferation and apoptosis, essential biological features of malignant tumors also include cell metastasis. Cancer metastasis is one of the major reasons causing cancer aggravation and mortality in gastric cancer patients [42, 43]. For instance, studies have demonstrated that matrix metalloproteinases (MMPs) altered their expressions in gastric cancer metastatic tumors, and they could be used as prognostic diagnostic markers in advanced gastric cancer patients as their up-regulation promoted caner metastasis in malignant tumors [44–46]. Therefore, more thorough studies are in need to explore the anti-tumor effects of germacrone, also to further elucidate its mechanisms of regulating gastric cancer. The regulations of all these important regulators by germacrone could be serving as promising therapeutic targets for gastric cancer.

## Conclusion

In conclusion, germacrone inhibits the proliferation of gastric cancer BGC823 cells by inducing the G2/M phase cell cycle arrest and apoptosis through regulation of cell cycle-associated proteins cyclin B1, cdc 2, and cdc 25c, and apoptosis-associated proteins procaspase-3, − 6, − 8, − 9, cleaved caspase-3, − 6, − 8, − 9 and cleaved PARP. This study provides insights into the application of germacrone in gastric cancer treatment.

## Data Availability

The analyzed data sets generated during the study are available from the corresponding author on reasonable request.
